The article "Suppression of NF-κB signaling by ECN in an arthritic model of inflammation" was retracted in 2023. Reasons: duplicated images; duplicated data; unreliable data; concerns about the data.

# Suppression of NF-κB signaling by ECN in an arthritic model of inflammation

**DOI:** 10.1186/s12906-022-03629-7

**Published:** 2022-06-13

**Authors:** Amna Khan, Li Zhang, Chang Hu Li, Ashraf Ullah Khan, Bushra Shal, Adnan Khan, Sajjad Ahmad, Fakhar ud Din, Zia ur rehman, Feng Wang, Salman Khan

**Affiliations:** 1 Pharmacological Sciences Research Lab, Department of Pharmacy, Faculty of Biological Sciences, Quaid-i-Azam University, Islamabad, Pakistan; 2 Department of Medical Oncology, Cancer Center, West China Hospital, West China Medical School, Sichuan University, Sichuan, People’s Republic of China; 3 Division of Radiation Physics, Cancer Center, West China Hospital, Sichuan University, Chengdu, 610041 Sichuan China; 4 Faculty of Pharmaceutical Sciences, Abasyn University, Peshawar, KPK Pakistan; 5 Department of Health and Biological Sciences, Abasyn University, Peshawar, 25000 Pakistan; 6 Department of Pharmacy, Faculty of Biological Sciences, Quad-i-Azam University, Islamabad, Pakistan; 7 Department of Chemistry, Quaid-I-Azam University, Islamabad, 45320 Pakistan

**Keywords:** Arthritis, Lipopolysaccharide, Immunomodulation, Inflammation, Oxidative stress

## Abstract

**Background:**

The 7β-(3-ethyl-*cis*-crotonoyloxy)-1α-(2-methylbutyryloxy)-3,14-dehydro-Z-notonipetranone (ECN), a sesquiterpenoid isolated from the *Tussilago farfara* Linneaus (Asteraceae), was evaluated against acute Carrageenan and chronic complete Freund’s adjuvant (CFA)-induced arthritis in mice.

**Methods:**

Acute and chronic arthritis were induced by administering Carrageenan and CFA to the intraplantar surface of the mouse paw. Edema, mechanical allodynia, mechanical hyperalgesia, and thermal hyperalgesia were assessed in the paw. Similarly, histological and immunohistological parameters were assessed following arthritis induced by CFA. Antioxidants, inflammatory cytokines, and oxidative stress markers were also studied in all the treated groups.

**Results:**

The ECN treatment significantly attenuated edema in the paw and elevated the nocifensive threshold following induction of this inflammatory model. Furthermore, ECN treatment markedly improved the arthritis index and distress symptoms, while attenuating the CFA-induced edema in the paw. ECN treatment also improved the histological parameters in the paw tissue compared to the control. At the same time, there was a significant reduction in edema and erosion in the ECN-treated group, as measured by radiographic analysis. Using the Comet’s assay, we showed that ECN treatment protected the DNA from chronic CFA-induced arthritis. Immunohistochemistry analysis showed a marked decrease in the expression level of p-JNK (phosphorylated C-Jun N-terminal kinase), NF-κB (Nuclear factor-kappa B), COX-2 (Cyclooxygenase-2), and TNF-α (Tumour necrosis factor-alpha) compared to the CFA-treated group. Biophysical analysis involving molecular docking, molecular dynamics simulations, and binding free energies of ECN were performed to explore the underlying mechanism.

The article "Suppression of NF-κB signaling by ECN in an arthritic model of inflammation" was retracted in 2023. Reasons: duplicated images; duplicated data; unreliable data; concerns about the data.

**Conclusion:**

ECN exhibited significant anti-inflammatory and anti-arthritic activity against Carrageenan and CFA-induced models.

**Supplementary Information:**

The online version contains supplementary material available at 10.1186/s12906-022-03629-7.

## Background

Rheumatoid arthritis (RA) is an autoimmune disorder characterized by synovial inflammation leading to articular destruction, joint stiffness, and pain [1]. It is one of the most prevalent disorders worldwide, affecting nearly 1–2% of the population [1]. The incidence of RA appears to be higher in people over 40 years of age and in women due to the loss of bone integrity after menopause [2]. The ultimate target of RA treatment includes alleviating inflammation, protecting articular morphology, maintaining physiology, and systemic control of mediators [3]. Treatment strategies for RA include non-steroidal anti-inflammatory drugs (NSAIDs), corticosteroids, and immunomodulators [4]. These agents help to lower arthritis-associated inflammation, but 30% of the individuals with RA fail to respond to the treatment [5]. Cost-effectiveness and reduced side effects are the primary parameters considered in the treatment of RA [2].

Complete Freund’s adjuvant (CFA) has been widely used to model RA in animals. It establishes autoimmune arthritis by increasing the inflammatory cytokines such as TNF-α, COX-2, and interleukin-1β (IL-1β) via NF-κB signaling [6–8]. CFA administration also induces activation of NF-κB by facilitating the degradation of IκB (inhibitory kappa B) [1, 9]. Following degradation of IκB, the NF-κB translocates to the nucleus and induces the expression of pro-inflammatory cytokines and oxidative stress markers [6–8]. Numerous experimental findings associated with the pathogenesis of arthritis reported that activation of NF-κB, along with conversion of superoxide anions to nitric oxide (NO) and reactive oxygen species (ROS) productionplay a major role in exaggerating arthritis [6–8]. These reactive oxygen species may also be involved in the paw tissue’s oxidative DNA damage, resulting in apoptosis [10]. In addition, some of the intracellular enzymes such as catalase (CAT), superoxide dismutase (SOD), glutathione (GSH), and glutathione sulfotransferase (GST) are detoxifying enzymes that may attenuate the pathological symptoms [11–13].

Phytochemicals have effectively alleviated or ameliorated numerous inflammatory disorders [14]. *Tussilago farfara* L. (Asteraceae), commonly called coltsfoot, is a perennial herb widely spread in Korea, China, North Africa, Siberia, and Europe [15]. The flowering buds of *T. farfara* have been used as an herbal medicine to treat asthma, bronchitis, and cough [15]. Several active sesquiterpenoids, such as faradiol, phytosterol, rutin, and tussilagone isolated from *T. farfara* possess anti-microbial and stimulate the cardiovascular system [16, 17].

The article "Suppression of NF-κB signaling by ECN in an arthritic model of inflammation" was retracted in 2023. Reasons: duplicated images; duplicated data; unreliable data; concerns about the data.

One of these is 7β-(3-ethylcis-crotonoyloxy)-1α-(2-methylbutyryloxy)-3,14-dehydro-Z-notonipetranone (ECN) known to have antioxidant and neuroprotective effects [15]. This study assessed the anti-arthritic activity of ECNagainst Carrageenan and CFA (augmented with LPS)-induced arthritis in mice to understand its possible molecular mechanism of anti-rheumatism.

## Methods

### Chemicals

ECN (the dried flower buds of *Tussilago farfara*) were purchased from an Oriental Market in Seoul, Korea, and identified by Prof. Je-Hyun Lee. Carrageenan, Complete Freund’s adjuvant (CFA), and Griess reagent were purchased from Sigma Aldrich (USA). ELISA kits for assessing the inflammatory mediators TNF-α and IL-1β were purchased from Thermo Fisher Scientific (USA). Primary and secondary antibodies were purchased from Santa Cruz. A Neubauer hemocytometer (Feinoptik, Germany) was used for blood analysis, while Sahli’s hemoglobin meter was used to measure the hemoglobin concentration (Hb). The AMP diagnostic kits (Graz, Austria) were utilized for the liver function tests. All the compounds were dissolved in 2% DMSO and then diluted with normal saline. All experiments were performed in triplicate to assess reproducibility.

### Plant material

The dried flower buds of *T. farfara* were purchased from Oriental Market in Seoul, Korea, and identified by Prof. Je-Hyun Lee (Dongkkuk University, Kyungju, South Korea). A voucher specimen (no. EA333) was deposited at Natural Product Chemistry Lab, College of Pharmacy, Ewha Womans University, Seoul, Korea) as reported [18].

### Animals

Male albino BALB/c mice (4–5 weeks of age; 25–30 g) were procured from the National Institute of Health (NIH), Islamabad, Pakistan. Animals were caged in a controlled laboratory environment with a room temperature of 23 ± 1 °C, 50 ± 10% humidity, and a 12 h light-dark cycle. The animals were provided unrestricted access to water and food. Procedures were carried out between 8 a.m. and 6 p.m. in the pathogens-free zone of the Pharmacology Laboratory, Department of Pharmacy, Quaid-i-Azam University, Islamabad, Pakistan. All experiments were performed following the guidelines of the ethical committee of Quaid-i-Azam University of care and experimental animals (Approval No: BEC-FBS-QAU2018–125) and conformed to the ethical instructions for the analysis of investigational pain in live animals developed by the International Association of Pain [19]. Great care was taken to avoid any unnecessary harm to the animals. New animals were used for each experiment and used once.

The article "Suppression of NF-κB signaling by ECN in an arthritic model of inflammation" was retracted in 2023. Reasons: duplicated images; duplicated data; unreliable data; concerns about the data.

### Randomization and sample size selection

Animals were randomly divided into various groups [20]. Double blindness was maintained during the whole experiment to avoid experimental biases. The sample size (*n* = 7) selection was based on previous reports [20].

### Animal models

Carrageenan-induced model: Mice were divided into six groups (*n* = 7 per group). The animals were divided randomly and equally into various groups to avoid scientific bias.

Group I: Normal control.

Group II: Carrageenan treated group (1% solution of Carrageenan, intraplantar).

Group III: Dexa 5 mg/kg, i.p. (60 min before Carrageenan administration).

Group IV: ECN 1 mg/kg, i.p. (60 min before Carrageenan administration).

Group V: ECN 5 mg/kg, i.p. (60 min before Carrageenan administration).

Group VI: ECN 10 mg/kg, i.p. (60 min before Carrageenan administration).

CFA-induced arthritis model: All the mice were allocated into four groups (*n* = 7 per group).

Group I: Normal control.

Group II: CFA treated group (20 μl, intraplantar).

Group III: Dexa 5 mg/kg, i.p. (forty min before CFA administration).

Group IV: ECN 10 mg/kg, i.p. (forty min before CFA injection).

Control animals received no treatment, the positive control received dexamethasone, and the treatment control regularly received ECN for 21 days. LPS (25 μg/kg, intraplantar) was also administered to all groups (except the control) on day 14 to augment the inflammatory response. The study design is depicted in Fig. 1.

**Fig. 1:** Study design of the ECN against the Carrageenan and CFA-induced models

### Animal sampling

Blood was obtained from the heart directly following anesthesia using xylazine and ketamine injection (16 mg + 60 mg, i.p). The animals were sacrificed by cervical dislocation [21].

#### Assessment of distress symptoms and survival rate in CFA -induced mice

Animals were observed throughout the experiment to assess the distress symptoms and survival rate in CFA- induced mice [22]. As reported previously, the assessed distress symptoms included general health, gait weakness, and unwillingness to move [22]. The distress score was calculated at different time intervals, i.e., 0, 3, 6, 9, 12, 15, 18, and 21st day [22]. Furthermore, the mortality rate was assessed in each group from day 0 to the end of the experiment.

The article "Suppression of NF-κB signaling by ECN in an arthritic model of inflammation" was retracted in 2023. Reasons: duplicated images; duplicated data; unreliable data; concerns about the data.

#### Assessment of arthritic score in CFA-induced mice

The structural characteristics of arthritis, such as redness, edema, and erythema, were assessed by the previously mentioned visual criteria [23]. A score of 0 indicatesno signs of redness and edema in the paw, 0.5 represents redness and swelling in just one finger, 1 indicates redness and light swelling of the ankle or 2–5 fingers, 2 indicates redness and medium swelling of the ankle and 2–5 fingers, 3 indicates redness and extreme swelling all fingers and 4 indicates decreased swelling and deformation resulting in an incapacitated limb.

#### Assessment of paw edema in Carrageenan and CFA-induced mice

The effect of ECN was assessed on Carrageenan and CFA-induced changes in paw thickness; the paw thickness was determined via dial thickness gauge [24, 25]. Paw edema was determined at four different time intervals in the case of Carrageenan and acute CFA-induced arthritis, i.e., 0, 2, 4, and 6 h. In the case of chronic CFA-induced arthritis, paw edema was determined on a daily basis for 21 days post-CFA administration .

#### Assessment of mechanical hyperalgesia in Carrageenan and CFA-induced mice

Paw withdrawal threshold in Carrageenan and CFA -induced mice were determined using the Randall Selitto apparatus (Digital Randall Selitto with Pressure Applicator) following published methods [5, 24]. The paw withdrawal threshold was determined on a daily basis for 21 days post-CFA.

#### Assessment of thermal hyperalgesia in Carrageenan and CFA-induced mice

Thermal pain threshold in Carrageenan and CFA-induced mice were determined using a unilateral hot plate apparatus [26]. The plate’s temperature was set at 50 ± 0.5 °C, and 35 seconds was set as a cut-off value to avoid the animal’s harm. The paw withdrawal latency was determined on a daily basis for 21 days post-CFA.

#### Assessment of mechanical allodynia in Carrageenan and CFA -induced mice

Mechanical allodynia was assessed using Von Frey filaments [11, 27, 28]. The paw withdrawal threshold was determined on a daily basis for 21 days post-CFA.

#### Estimation of GSH, GST, CAT, and SOD in CFA-induced mice paw tissue

The effect of ECN (10 mg/kg, i.p) on the antioxidants GSH, GST, CAT, and SOD was determined as reported previously [29–31]. Briefly, the reduced glutathione was assessed by mixing tissue homogenate (0.1 ml), PBS solution (2.4 ml), and DTNB (0.5 ml) to make the final volume up to 3 ml. The absorbance was read by a microplate reader at 412 nm wavelength. The GST level was quantified following the previously mentioned method [28–30]. The GST level in paw tissue was assessed by mixing tissue homogenate (0.1 ml), CDNB (0.1 ml), and by adding 0.1 M PBS (pH 6.5) to make the final volume of 3 ml. The absorbance was read by a microplate reader at a wavelength of 314 nm. Catalase level was analyzed following the already mentioned protocol with minor adjustments [22]. The catalase level was assessed by taking H_2_O_2_-phosphate buffer (3 ml) in a cuvette and by rapid addition of enzyme extract (40 μl) [31]. The absorbance was read by a microplate reader at 240 nm wavelength. The SOD activity was measured by mixing 50 mM (pH 8.5) Tris-EDTA buffer, 24 mM pyrogallol, and 10 μl of the sample [31]. The absorbance was read at 420 nm wavelength.

The article "Suppression of NF-κB signaling by ECN in an arthritic model of inflammation" was retracted in 2023. Reasons: duplicated images; duplicated data; unreliable data; concerns about the data.

#### Estimation of NO and MDA in CFA-induced plasma

Nitric oxide (NO) levels in CFA -induced mice paw tissue were assessed via the Griess reagent method, as reported [24, 32]. Similarly, the rate of lipid peroxidation was analyzed by assessing the concentration of malonaldehyde (MDA) [29, 30]. Briefly, tissue homogenate (0.25 ml) in 10% PBS (pH 7.4) was incubated at 37 °C in a water bath. After 1 h incubation, 5% TCA (0.25 ml) and 0.67% TBA (0.5 ml) were mixed with the tissue homogenate (0.25 ml) and centrifuged at 1300 rpm for 10 min. The clear supernatant was transferred from the above mixture to a different tube, placed for 10 min in a water bath, cooled, and the absorbance read at 535 nm wavelength.

### Detection of inflammatory cytokines

Production of TNF-α and IL-1β following CFA-induced arthritis was measured using ELISA kits. Briefly, the paw tissue samples from all the animal groups were prepared according to method described above. Protein was extracted from the tissue using PBS \ with 0.4 M NaCl, 0.05% Tween 20, and protein inhibitors. The samples were homogenized and centrifuged (at 3000 g for 10 min) to obtain the supernatant for the assessment of the TNF-α and IL-1β using commercially available kits [33].

#### Estimation of DNA damage in CFA-induced mice paw tissue

DNA damage was assessed by comet assay [34, 35]. A small part of the paw tissue was suspended in cold lysing buffer (1 ml) in an ultracentrifuge tube, and then the samples were homogenized. The cell suspension (5–10 μl) was mixed in 0.5% low melting point agarose, layered on the pre-coated slides with normal agarose solution (1%), and incubated for 10 min on an ice pack. After performing this step twice, the slides were placed in lysing mixture for 2 h at 4 °C. Post-electrophoresis, slides were marked with ethidium bromide (1%) and were analyzed under a fluorescent microscope. The content of DNA disruption was quantified by CASP software. Length of tail and % DNA in the tail was used to check DNA disruption’s content [34, 35].

### Renal and hepatotoxicity testing

The effect of ECN (10 mg/kg, i.p) treatment on the vital organs such as the liver and kidneys was assessed by measuring the aspartate aminotransferase (ALT), alanine aminotransferase (AST), and creatinine concentration [21]. The collected blood was centrifuged at 5000 rpm for 5 min to separate the plasma from the blood. The plasma was used to estimate the concentration of AST, ALT, and creatinine [21].

The article "Suppression of NF-κB signaling by ECN in an arthritic model of inflammation" was retracted in 2023. Reasons: duplicated images; duplicated data; unreliable data; concerns about the data.

#### Radiological and histological analysis

Radiological analysis was carried out to assess ECN (10 mg/kg) treatment on synovial hyperplasia, tissue and joint destruction following CFA-induced arthritis, as mentioned [21]. Radiographic images of all the groups were taken and quantified using the digital radiographic system, as reported [6]. H and E staining assessed the underlying histopathological changes following CFA-induced arthritis. The paw tissue was placed in formalin solution (10%), mounted in paraffin blocks, sliced into 4 μm sections, and observed under a microscope (100X) [6].

#### Hematological analysis

Blood was analyzed for total leukocyte count, different leukocytes, and erythrocytes in all the animal groups [6].

### Immunohistochemical expression of TNF-α, COX-2, p-JNK, and p-NF-κB in CFA-induced mice paw tissue

Immunohistochemical analysis of TNF-α, COX-2, p-JNK, and p-NF-κB was performed according to the published method [22]. Briefly, paw tissues (paraffin-fixed) were deparaffinized and rehydrated through xylene and alcohol. The intracellular peroxidase was quenched by H_2_O_2_ (3%) in menthol and then incubated for 20 min with goat serum. The slides were incubated overnight with mouse anti-TNF-α, anti-COX-2, anti-p-JNK, and anti-NF-κB antibodies [36]. After washing, the slides were incubated in secondary antibodies (goat-antimouse), then incubated with ABC reagents for 1 h,washed with phosphate buffer saline and marked with diaminobenzidine solution. Images were taken under a light microscope. The relative expression of TNF-α, COX-2, p-JNK, and NF-κB was measured using Image_J software [37].

#### Molecular docking analysis

Computational analysis is commonly employed to assess the interaction of the ligand with the protein targets and explore the mechanism of binding of the ligand with the protein [37]. In the present study, the molecular docking analysis of ECN against the various targets was performed using AutoDock Vina 4.2. The protein targets were downloaded from the RCSB PDB site (RCSB.PDB) and saved in PDB format. The water molecules and co-crystallized ligands were removed during protein preparation, and the energy was minimized [37]. The ligand was prepared using chembiodraw_16 and saved as an SDF file. The SDF file was converted to PDB format, and the ligand’s energy was minimized [37]. The binding energies and interacting amino acids with the ligands were represented in 3D and 2D structures.

The article "Suppression of NF-κB signaling by ECN in an arthritic model of inflammation" was retracted in 2023. Reasons: duplicated images; duplicated data; unreliable data; concerns about the data.

### Molecular dynamics simulation

The stable energy ECN-JNK and ECN-p65 complexes were further investigated for structural stability and estimation of binding free energies. Molecular Dynamic simulation was performed on NVIDIA GPU RTX1080 TI using Particle Mesh Ewald Molecular Dynamics (PMEMD.CUDA) from AMBER20. Initially, the complex was processed by employing Antechamber and the FF14SB force field [37, 38]. The latter was considered to define molecular characteristics and generate coordinate and topology files. Each complex was then solvated in a TIP3P water box, and subsequently, counter ions were added to obtain neutral systems. A production run was performed for 200 ns under periodic boundary conditions for each system. SHAKE algorithm was used to allow constraints on bonds containing hydrogen while long-range electrostatic interactions were processed through Particle Mesh Ewald (PME) method [37, 38]. Prior, systems energy was equilibrated and gradually increased to 300 K for 100 ps with additional 500 ps constant number of particles, pressure, temperature (NPT) equilibration, and pressure 1 atm. The production run of MD via steepest descent and conjugate gradient methods. In the heating step, systems temperature simulation was performed without any constraints for the timescale of 200 ns. The MD simulation trajectories were analyzed through the CPPTRAJ program of AMBER. The MMPBSA.py was consequently used to estimate binding free energy based on Molecular Mechanics-Poisson Boltzmann Surface Area (MM-PBSA) method [37, 38].

#### Pharmacokinetic analysis

The pharmacokinetic parameter of the ECN was assessed using computational analysis as reported previously [37, 38]. The parameters that were assessed during the current studies include absorption, metabolism, distribution, and excretion using Swiss target predictions (www.swisstargetprediction.com), pkCSM (biosig.unimelb .edu.au/pkcsm/prediction), and PASS online (www.pharmaexpert.ru/passonline/) [38]. Furthermore, the physico-chemicals properties such as water solubility, lipid solubility, number of rotational bonds, hydrogen donor/acceptor, and drug-likeness behavior were assessed [38]. The possible metabolites of ECN were predicted using GLORY metabolites software (https://nerdd.zbh.uni-hamburg.de/glory/about/) and were ranked according to the possibility of their occurrence [38].

#### Statistical analysis

The values are expressed as mean ± S. D (*n* = 7) and evaluated using a one-way analysis of variance (ANOVA) followed by the post hoc test to assess the inter-group comparisons, while two-way repeated analysis of variance (ANOVA) was used where appropriate. *P*-values such as *p* < 0.05, *p* < 0.01, and *p* < 0.001 were considered significant. GraphPad Prism version_5 was used for the statistical analysis.

The article "Suppression of NF-κB signaling by ECN in an arthritic model of inflammation" was retracted in 2023. Reasons: duplicated images; duplicated data; unreliable data; concerns about the data.

## Results

### Effect of ECN on Carrageenan-induced paw edema, thermal hyperalgesia, mechanical hyperalgesia, and mechanical allodynia

Carrageenan-induced paw edema was used as a preliminary model to investigate the effect of ECN and optimize the dose-response. The ECN treatment was evaluated in different concentrations (1 mg/kg, 5 mg/kg, and 10 mg/kg) against paw edema, mechanical hyperalgesia, mechanical allodynia, and thermal hyperalgesia induced by Carrageenan. ECN markedly reduced paw edema compared to the Carrageenan-induced group (*p* < 0.05). The dose of 10 mg/kg exhibited the maximum response. Similarly, ECN attenuated the mechanical hyperalgesia (*p* < 0.01) and allodynia (*p* < 0.05) while significantly increasing the pain threshold compared to the Carrageenan-induced group. Furthermore, ECN administration significantly reduced the acute Carrageenan-induced thermal hyperalgesia (p < 0.05) and increased the pain threshold compared to the Carrageenan-induced group, as shown in Fig. 2. The ECN dose of 10 mg/kg was optimal and used in subsequent experiments.

**Fig. 2:** The effect of ECN (1, 5, and 10 mg/kg) on the acute carrageenan-induced edema. ECN (1, 5, and 10 mg/kg) inhibited (**A**) paw edema (**B**) thermal hyperalgesia (**C**) mechanical hyperalgesia, and (**D**) mechanical allodynia. The data were represented as the mean ± SD (*n* = 7). (*) *p* < 0.05, (**) *p* < 0.01 and (***) *p* < 0.001 indicates significant differences from the CFA control group, while (###) means comparison with the CFA treated group

### Effect of ECN on CFA-induced survival rate, distress symptoms, and arthritic index

CFA-induced arthritis is associated with the development of distress symptoms in animals [33]. CFA showed a marked increase in the distress symptoms. However, ECN administration showed remarkable improvement in the distress symptoms. Similarly, CFA showed a marked increase in the arthritic index (inflammation of the joints, number of inflamed digits, and erythema). However, the ECN exhibited a marked reduction in the arthritic index compared to the CFA-induced group (*p* < 0.01). Furthermore, survival analysis showed no significant changes in the mortality rate of any treated group (Fig. 3).

**Fig. 3:** Effect of ECN treatment on survival rate, distress symptoms, and arthritic index. **A** Survival rate showed no significant difference amongst the studied groups. **B** The ECN showed significant improvement in the distress symptoms (Dull/Ruffled coat, change in temperament, reluctance to move) compared to the CFA treated group. **C** Furthermore, the ECN treatment markedly improved the arthritic score in contrast to CFA treated group. The data were represented as the mean ± SD (*n* = 7). (*) *p* < 0.05, (**) *p* < 0.01 and (***) *p* < 0.001 indicates significant differences from the CFA control group, while (###) means comparison with the CFA treated group

The article "Suppression of NF-κB signaling by ECN in an arthritic model of inflammation" was retracted in 2023. Reasons: duplicated images; duplicated data; unreliable data; concerns about the data.

### Effect of ECN on CFA-induced paw edema and thermal hyperalgesia

The CFA -induced group showed an increase in paw edema in both acute and chronic models. However, ECN administration reduced paw swelling compared to the CFA-induced group (*p* < 0.05) (Fig. 4). The thermal hyperalgesia threshold in acute and chronic studies was significantly decreased in the CFA-induced group. However, ECN increased the thermal hyperalgesia threshold compared to the CFA-induced group (*p* < 0.01) (Fig. 4).

**Fig. 4:** The effect of the ECN (10 mg/kg) treatment on the CFA-induced paw edema and thermal hyperalgesia. The ECN markedly attenuated the CFA-induced both acute paw edema (**A**) and chronic paw edema (**B**) compared to the CFA treated group. Similarly, the ECN treatment showed marked increase in the thermal hyperalgesic responses in both acute (**C**) and chronic (**D**) models as compared to the CFA treated group. The data were represented as the mean ± SD (*n* = 7). (*) *p* < 0.05, (**) *p* < 0.01 and (***) *p* < 0.001 indicates significant differences from the CFA control group, while (###) means comparison with the CFA treated group

### Effect of ECN on CFA-induced mechanical hyperalgesia and allodynia

The CFA administration significantly reduced the mechanical hyperalgesia threshold in acute and chronic studies, while this was significantly increased following treatment with ECN (*p* < 0.05) (Fig. 5). Similarly, the CFA-induced group showed a marked decrease in the mechanical allodynic threshold in acute and chronic studies which was significantly enhanced ECN (Fig. 5).

**Fig. 5:** Effect of the ECN (10 mg/kg) on the mechanical hyperalgesia and mechanical allodynia following CFA-induced arthritis. The ECN treatment marked improved hyperalgesic responses (**A**, **B**) when compared to CFA treated group. Similarly, the ECN treatment attenuated the allodynia (**C**, **D**) significantly in both acute and chronic models compared to control. The data were represented as the mean ± SD (*n* = 7). (*) *p* < 0.05, (**) *p* < 0.01 and (***) *p* < 0.001 indicates significant differences from the CFA control group, while (###) means comparison with the CFA treated group

The article "Suppression of NF-κB signaling by ECN in an arthritic model of inflammation" was retracted in 2023. Reasons: duplicated images; duplicated data; unreliable data; concerns about the data.

### Effect of ECN on antioxidant proteins and enzymes in CFA-induced mice paw tissue

CFA-induced arthritis is associated with increased oxidative stress (MDA, NO) and reduction in the antioxidants GSH, GST, Catalase, and SOD. In the present study, there was a reduction in the antioxidants GSH, GST, Catalase, and SOD and a marked increase in the oxidative stress markers MDA and NO. ECN treatment resulted in an increase (*p* < 0.001) in the antioxidantsand a significant reduction (*p* < 0.001) in the MDA and NO levels compared to the CFA-induced group (Fig. 6).

**Fig. 6:** Effect of ECN (10 mg/kg) on the antioxidants and oxidative stress markers in the CFA-induced model. **A** ECN treatment promisingly enhanced the antioxidants level such as (**A**) GSH, (**B**) GST, (**C**) SOD and (**D**) Catalase compared to the CFA treated group. Furthermore, the ECN treatment also significantly attenuated the oxidative stress markers such as (**E**) NO and (**F**) MDA in comparison to CFA treated group. The data were represented as the mean ± SD (*n* = 7). (*) *p* < 0.05, (**) *p* < 0.01 and (***) *p* < 0.001 indicates significant differences from the CFA control group, while (###) means comparison with the CFA treated group

### Effect of ECN on pro-inflammatory cytokines

CFA administration elevated the levels of IL-1β and TNF-α in the paw tissue measured by ELISA; this effect was reversed by ECN (Fig. 7). Likewise, CFA significantly increased the expression of TNF-α, COX-2, p-JNK, and p-NF-κB measured by immunohistochemistry (Fig. 8X). ECN reduced the expression level of these proteins compared to the CFA treated group.

**Fig. 7:** The influence of the ECN on the inflammatory cytokines such as TNF-α (**A**) and IL-1β (**B**) following CFA-induced arthritis. The CFA-treated group showed a marked increase in the level of the pro-inflammatory cytokines. However, the ECN showed a marked reduction in the inflammatory cytokines compared to the CFA (sensitized with the LPS)-induced group. The data were represented as the mean ± SD (*n* = 7). (*) *p* < 0.05, (**) *p* < 0.01 and (***) *p* < 0.001 indicates significant differences from the CFA control group, while (###) means comparison with the CFA treated group

**Fig. 8:** Effect of ECN (10 mg/kg) treatment on expression of TNF-α, COX-2, p-JNK, and NF-κB using immunohistochemical analysis (scale bar = 100 μm). The ECN treatment showed significant attenuation of the TNF-α, COX-2, p-JNK, and NF-κB expression levels following CFA treated group. The images were taken at 10X using a simple microscope attached to the camera. Representative images are 10X original magnification are reflecting activation of TNF-α, COX-2, p-JNK, and NF-κB. The data were represented as the mean ± S.D. (*n* = 7). (*) *p* < 0.05, (**) *p* < 0.01 and (***) *p* < 0.001 indicates significant difference from the CFA control group, while (###) means comparison with the CFA treated group

The article "Suppression of NF-κB signaling by ECN in an arthritic model of inflammation" was retracted in 2023. Reasons: duplicated images; duplicated data; unreliable data; concerns about the data.

### Effect of ECN on kidney and liver functions

Changes in liver and kidney functions were assessed by determining ALT, AST, and creatinine levels in all the animal groups following CFA-induced arthritis. Daily ECN treatment for 21 days had no effect on the liver and kidney markers (AST, ALT, and creatinine) (Table 1).

**Table 1:** Effect of the ECN (10 mg/kg) on hematological parameters such as total WBCs count, differential WBCs count, and RBCs level following CFA-induced arthritis

Parameters	WBC (10^**9**^/L)	LYM (10^**9**^/L)	NEU (10^**9**^/L)	MON (10^**9**^/L)	RBC (10^**12**^/L)	PLT (10^**9**^/L)
**Normal control**	3.8 ± 0.18	2.02 ± 0.06	0.40 ± 0.029	0.32 ± 0.015	5.42 ± 0.3	257 ± 12
**CFA**	5.33 ± 0.12^**###**^	3.6 ± 0.17^**###**^	0.71 ± 0.18^**###**^	0.54 ± 0.16^**###**^	5.63 ± 0.29^**###**^	113 ± 22^**###**^
**ECN (10 mg/kg)**	3.96 ± 0.24	2.26 ± 0.11	0.54 ± 0.056	0.38 ± 0.045	5.84 ± 0.12	205 ± 15

The results showed no significant changes in the hematological parameters in all the treated groups. The data were represented as the mean ± SD (*n* = 7). (*) *p* < 0.05, (**) *p* < 0.01 and (***) *p* < 0.001 indicates significant differences from the CFA control group, while (###) means comparison with the CFA treated group

### Effect of ECN on radiological and histological examination

Radiological analysis was performed to assess the changes in the paw tissue and subsequently assess the effect of ECN following CFA-induced arthritis [39]. CFA administration resulted in an increase in soft tissue swelling, cartilage destruction, synovial hyperplasia, and bone erosion [39]. In contrast, ECN reduced paw swelling, synovial hyperplasia, and bone erosion (Fig. 9). By H&E staining, CFA induced a significant increase in immune cell infiltration, paw edema, and changes in histological architecture. ECN (10 mg/kg) treatment showed marked improvement in the histological features compared to the CFA-induced group (*p* < 0.01) (Fig. 9).

**Fig. 9:** Effect of ECN on radiological and histological examination (scale bar = 100 μm) following CFA-induced arthritis. The ECN improved the radiological parameters such as soft tissue swelling compared to the CFA treated group. The radiological changes in all the recruited groups were quantified in all the treated groups. Similarly, the H and E staining showed marked improvement in the histological parameters such as synovial hyperplasia, destruction of cartilage/bone and inflammatory cell infiltrate. The pathological changes were quantified as described in the “Materials and methods” section. The images were taken at 100X using a simple microscope attached to the camera. The data were represented as the mean ± SD (*n* = 7). (*) *p* < 0.05, (**) *p* < 0.01 and (***) *p* < 0.001 indicates significant differences from the CFA control group, while (###) means comparison with the CFA treated group

The article "Suppression of NF-κB signaling by ECN in an arthritic model of inflammation" was retracted in 2023. Reasons: duplicated images; duplicated data; unreliable data; concerns about the data.

### Effect of ECN on DNA damage in paw tissue

The Comet assay was performed to assess changes to DNA in the paw tissue [39]. We observed marked changes in the DNA integrity, including DNA tailing and % DNA in the tail in response to CFA. ECN preserved the DNA architecture (DNA tailing and % DNA in tail) compared to the CFA-induced group (*p* < 0.05) (Fig. 10).

**Fig. 10:** Effect of ECN (10 mg/kg) on DNA damage in paw tissue analyzed by comet assay (scale bar = 100 μm). Fluorescence photomicrographs showed significant protection of the DNA following CFA treated group in the paw tissue. The changes in the DNA content were estimated by tail length and % DNA in the tail in all the treated groups. The data were represented as the mean ± SD (*n* = 7). (*) *p* < 0.05, (**) p < 0.01 and (***) *p* < 0.001 indicates significant difference from the CFA control group, while (###) means comparison with the CFA treated group

### Effect of ECN on hematological changes

Changes in the levels of RBCs, total leukocytes count, and differential leukocytes count (neutrophils, eosinophils, platelets, and monocytes) were measured in all the recruited groups. The hematological studies revealed no significant changes in the hematological parameters (Table 2).

**Table 2:** Effect of ECN (10 mg/kg) on the liver and renal function test following CFA-induced arthritis

Parameters	ALT (IU/L)	AST (IU/L)	Creatinine (mg/dl)
Normal control	25.33 ± 0.57	21.33 ± 0.57	1.09 ± 1.73
CFA	37.33 ± 1.52^**###**^	35.66 ± 3.51^**###**^	1.50 ± 4.04^**###**^
ECN (10 mg/kg)	30.81 ± 4.35	25.5 ± 2.64	1.20 ± 0.57

The results revealed no marked changes in the LFTs and RFTs in any group. The data were represented as the mean ± SD (*n* = 7). (*) *p* < 0.05, (**) *p* < 0.01 and (***) *p* < 0.001 indicates significant differences from the CFA control group, while (###) means comparison with the CFA treated group

### Molecular docking analysis

Molecular docking analysis was performed to assess the interaction of ECN with the protein targets JNK (PDB ID = 1uki), NF-κB (PDB ID = 1vkx), COX-2 (PDB ID = 1pxx), and TNF-α (PDB ID = 2az5). ECN showed variable interaction with the protein targets via multiple hydrophobic and hydrophilic bonds. The grid dimension center and size was maintained at (x = − 18.625, y = 74.475, z = 42.058) and (x = 100, y = 100, z = 100), respectively. The interaction of the ligand-receptor complex was visualized using Discovery studio visualizer_16, and the 3D and 2D images are shown in Fig. 11. ECN showed multiple hydrogen bonds and hydrophobic bonds with p65 (His 58A, Ser 112A, Thr 60A). Similarly, ENC also showed multiple hydrogen bonds with JNK (Arg 125A), COX-2 (His 2382C, Asn 2214C), and TNF-α (Tyr 151A). The negative binding energies of ECN with p65, JNK, COX-2, and TNF-α, as well as the interacting amino acids involved, are described in Table 3.

The article "Suppression of NF-κB signaling by ECN in an arthritic model of inflammation" was retracted in 2023. Reasons: duplicated images; duplicated data; unreliable data; concerns about the data.

**Fig. 11:** Molecular docking analysis of the ECN against the protein targets such as p-JNK, NF-κB, COX-2, and TNF-α. The molecular docking analysis showed interaction with the ECN via multiple hydrophilic and hydrophobic bonds. The interaction between the ligand and protein complex is shown in 3D and 2D views

**Table 3:** The interaction of the ECN with various protein targets using molecular docking analysis

Ligand-protein interaction	Binding energy (Kcal/mol)	Hydrogen bonds	Hydrogen bond amino acids	Hydrophobic interactions
ECN-JNK	−6.0	1	Arg25	Leu363, Leu23, Lys24, Asn9, Ala510
ECN-NF-κB	−6.0	3	His58, Ser112, Thr60	Ile110
ECN-COX-2	−7.4	2	His2212, Asn2382	Phe2210, His2207, Val2442, Ala2450, His2388, His2386, Ala2446
ECN-TNF-α	−8.1	1	Tyr151	Leu57, Tyr59, Tyr119

The molecular docking analysis showed multiple H-bonds and hydrophobic bonds of the ECN with various protein targets such as JNK, NF-κB, COX-2, and TNF-α. Additionally, the molecular docking analysis also showed the binding energies of the ECN with various protein targets and the amino acid involved in the interaction

### Molecular dynamics simulation

The binding stability of the ECN-JNK complex and ECN-p65 complex was explored by a run of molecular dynamics simulation for 200 ns. To investigate the intermolecular conformation and stability of interactions between the compounds and protein, root means square deviation (RMSD) analysis was performed using molecular dynamics simulation trajectories. RMSD measures the mean distance of superimposed protein atoms for a given simulation frame relative to a selected reference snapshot. Considering the RMSD plot for the ECN-JNK complex and ECN-p65 complex, both complexes attain sustainable structure conformational stability as the simulation proceeds (Fig. 12). The RMSD value of complexes throughout simulation time is within an acceptable range and depicts a highly stable nature. The ECN-p65 system, in particular, was reported to be more structurally stable due to strong hydrogen bonding with residues like His58 and Thr60. These interactions are seen regularly in interactions with the ECN compound and play a critical role in holding the ligand at the docked site. The initial RMSD deviations of the ECN-JNK complex correspond to ECN conformational moves. This suggests that the compound binding pose predicted by docking studies is not real, and the binding mode is subjected to conformational changes to make its interaction strength with active residues at the active site of JNK protein. Equilibrium of this complex can also be visualized after 100 ns, and this stability is stronger towards the end of the simulation. The mean RMSD of ENC-p65 and ECN-JNK complex is 1.40 Å and 1.69 Å, respectively.

The article "Suppression of NF-κB signaling by ECN in an arthritic model of inflammation" was retracted in 2023. Reasons: duplicated images; duplicated data; unreliable data; concerns about the data.

**Fig. 12:** RMSD plot of complexes based on carbon alpha atoms

### MMPBSA binding free energies

The MMPBSA binding free energy was estimated to affirm the docking and simulation results. From the data in Table 4, both systems are highly stable by acquiring highly negative total binding energy in kcal/mol. The overall binding free energy of ECN-JNK complex and ECN-p65 is − 44.38 kcal/mol and − 53.27 kcal/mol, respectively. The latter system, by binding energy, is more stable than the formal one. This net binding energy suggests the protein-ligand interactions are dominated by electrostatic energy and is equally supported by van der Waals energy. On the other hand, the non-polar biding energy like gas-phase energy favors complex formation, whereas negative contribution was reported from polar solvation energy.

**Table 4:** MMPBSA binding free energy of complexes in kcal/mol using a molecular dynamics simulation approach

Complex	Net Binding Free Energy	Net Electrostatic Binding Energy	Net van der Waals Binding Free Energy	Net Gas Phase Binding Energy	Net Polar Solvation Binding Free Energy	Net Non- polar Solvation Binding Free Energy	Net Solvation Binding Free Energy
ECN-JNK	−44.38	−25.99	−21.04	−47.03	11.78	−9.13	2.65
ECN-p65	−53.27	−35.64	−18.66	−54.3	8.00	−6.97	1.03

The MD simulation was performed for the NF-kB (p65) and JNK using AMBER20. The MD simulation showed various parameters such as net binding free energies, net electrostatic binding free energy, net van der Walls free energy, net gas phase binding energy, net polar solvation binding free energy, and net non-polar solvation binding free energy, and net solvation binding free energy

### Pharmacokinetic analysis

Pharmacokinetic parameters such as ADME (absorption, distribution, metabolism, and excretion), toxicokinetics, and physicochemical properties of the ECN were studied using an *in silico* approach. The absorption parameters included water-solubility, Caco2 cell permeability, intestinal absorption, P-glycoprotein inhibition, and P-glycoprotein substrate. Similarly, the distribution includes a volume of distribution (VDss), blood-brain barrier permeability, and fraction of unbound drug. The metabolism includes cytochrome p450 inhibition, while the excretion includes total clearance. The toxicokinetic parameters include Ames toxicity, hepatotoxicity, hERG I and II inhibition, and minnow toxicity. The drug-likeness behavior of ECN and various rules of the drug-likeness such as Lipinski, Ghose, Veber, Egan, and Muegge were assessed (Fig. 13). Similarly, the metabolites of ECN were predicted using a computational tool and were ranked according to the possibility of their occurrence (Fig. 14).

The article "Suppression of NF-κB signaling by ECN in an arthritic model of inflammation" was retracted in 2023. Reasons: duplicated images; duplicated data; unreliable data; concerns about the data.

**Fig. 13:** The pharmacokinetic parameters assessment of the ECN using *in silico* approach. The various parameters that were retrieved include absorption, metabolism, distribution, and excretion. Furthermore, the study also assesses the Physico-chemical parameters such as lipophilicity, hydrophobicity, rotational bonds, hydrogen donor/acceptor, and drug-likeness properties. The study also assesses the toxicokinetics parameters of the ECN against various organs and models

**Fig. 14:** The predicted metabolites of the ECN using the computational tool. The possible metabolites of the ECN were predicted based on the software previously similar compounds and assessing the structure of the ECN. The metabolites were ranked according to the obituary score generated by the software

## Discussion

Inflammation is a multidimensional biochemical and defensive process comprised of vascular permeability and nonspecific responses stimulated by the innate immune system to infection, injured cells, and irritants [40]. Histamine, serotonin, bradykinin, and prostaglandin are the important endogenous mediators critically involved in inflammation [41]. The Carrageenan-induced inflammatory event takes place in two phases. During the first phase, the various mediators of inflammation such as bradykinin, complement, and tachykinin are released; while in the second phase, there is a release of prostaglandins and other enzymes [42].

The CFA-induced model is commonly used to assess the chronic inflammatory microenvironment within arthritic inflammation and assess the mediators involved in the ongoing inflammatory process [43]. The pro-inflammatory mediators unleashed during the inflammatory event sensitize the pain receptors that cause inflammatory pain. All types of inflammatory pain are due to sensitization of primary nociceptive neurons, which results in hyperalgesia and allodynia [44, 45].

Currently, various strategies are used in clinical practice to deal with rheumatoid arthritis, including the NSAIDs (non-steroidal anti-inflammatory drugs), DMARDs (disease-modifying anti-rheumatic drugs), and biological drugs [46, 47]. However, these drugs are associated with various unavoidable adverse outcomes that necessitate drug abstinence. The NSAIDs are associated with gastric ulceration and cardiovascular adverse events [46, 47], while the biological and DMARDs are associated with immunosuppression and increased chance of infection. Given this, there is an urgent need to develop drugs that are safe and effective against rheumatoid arthritis. In the current study, ECN was assessed against Carrageenan and CFA-induced arthritis*.* ECN administration significantly increased paw withdrawal threshold and paw withdrawal latency in Carrageenan and CFA-induced mice.

The article "Suppression of NF-κB signaling by ECN in an arthritic model of inflammation" was retracted in 2023. Reasons: duplicated images; duplicated data; unreliable data; concerns about the data.

The histological studies play a key role in assessing the pathological changes within the inflammatory environment, such as infiltration of the inflammatory cells, edema, and fibrotic changes [48, 49]. Similarly, the radiological analysis assesses joint damage, stiffness, and inflammation [50, 51]. In the present study, ECN treatment significantly improved the histological and radiological features compared to the control. Other studies also reported that improvement in histological parameters of the paw tissue reduces inflammatory arthritis [46, 52].

Oxidative stress exacerbates the inflammatory process and is critically involved in the pathogenesis of rheumatoid arthritis [9]. The free radicals generated during the inflammatory process interact with cellular proteins, DNA, and lipids [9]. Free radicals such as superoxide and peroxides lead to the production of nitric oxide and MDA, which induce the production of pro-inflammatory mediators [53]. The body possesses the endogenous antioxidants system such as GST, GSH, Catalase, and SOD, which trigger the neutralization of the free radicals [25, 53]. CFA administration is commonly associated with alleviating the antioxidants and elevating oxidative stress markers [54]. In the current study, ECN significantly attenuated the oxidative stress markers and induced the antioxidants compared to the CFA treated group. The result of the current study is consistent with previously reported studies in which the reduction in oxidative stress and increase in the antioxidant showed amelioration of rheumatoid arthritis [52].

The increased activity of NF-κB signaling induces the production of numerous pro-inflammatory cytokines such as TNF-α, COX-2, and other biologically active substances [21]. COX-2, a critical pro-inflammatory mediator, triggers prostaglandin synthesis and accelerates the inflammatory process [13]. Similarly, MAPK (JNK) also regulates the synthesis of pro-inflammatory mediators, and its activation augments the inflammatory process [55, 56]. In the present study, ECN treatment markedly attenuated the expression levels of the pro-inflammatory proteins TNF-α, p-JNK, COX-2 and NF-κB compared to the CFA-treated group. Several other studies reported that inhibition of inflammatory cytokines such as TNF-α and COX-2 attenuates rheumatoid arthritis and improves the patient’s quality of life [57]. Additionally, activation of the MAPKs (JNK) and NF-κB signaling aggravate the underlying condition, while attenuation of NF-κB and MAPKs (JNK) reduce the signs and symptoms associated with rheumatoid arthritis [57].

The article "Suppression of NF-κB signaling by ECN in an arthritic model of inflammation" was retracted in 2023. Reasons: duplicated images; duplicated data; unreliable data; concerns about the data.

Quantitative DNA damage in paw tissue was identified by DNA relocation out of the nucleus and into the Comet’s tail. DNA strand breakage can be due to the enhanced generation of ROS, leading to free radical formation, which might be the reason for the alteration and strand breakage of double-helical strands causing cell death [34, 58]. Treatment with ECN remarkably reduced DNA damage compared to the CFA treated group.

Computational analysis has played a key role in developing and screening new drugs for the ailment of various diseases. Virtual screening is now being widely used to elucidate the possible mechanism of the drug against various targets [34]. In the present study, molecular docking analysis, molecular dynamics simulation, and MMPBSA binding free energy were performed to assess the binding affinity of ECN and its mechanism of interaction with the protein targets TNF-α p-JNK, COX-2, and NF-κB [34]. ECN had different binding energies and affinities for the protein targets; however, ECN exhibited a strong affinity for NF-κB and MAPKs (JNK). Based on the molecular docking binding energies, the ECN-NF-κB and ECN-JNK complexes were subjected to molecular dynamics simulation to assess the stability of the ligand-protein complexes and binding free energies. The ECN-NF-κB and ECN-JNK complexes showed RMSD values in the acceptable range, and the complexes remained stable during the simulation process. Similarly, the present computational analysis results are consistent with the previously reported studies [37, 38, 59, 60, 61].

## Conclusion

The present study investigated the anti-rheumatic potential of the natural compound ECN against Carrageenan and CFA-induced arthritis. ECN administration improved the signs and symptoms associated with acute and chronic inflammatory arthritis, including paw edema and pain. ECN administration restores the antioxidant and oxidative stress imbalance while significantly attenuating the inflammatory cytokines involved in the pathogenesis of rheumatoid arthritis. Furthermore, ECN treatment improved radiological and histological parameters by attenuating NF-kB and MAPKs (JNK) signaling and preserving DNA integrity. Similarly, ECN portrayed various physico-chemical properties and showed no toxicity against vital organs using computational and *in vivo* approaches. Overall, this study provides scientific evidence of ECN activity against inflammation and rheumatic arthritis. However, additional studies should be carried out to understand the mechanism of actionof ECN against Rheumatoid Arthritis.

The article "Suppression of NF-κB signaling by ECN in an arthritic model of inflammation" was retracted in 2023. Reasons: duplicated images; duplicated data; unreliable data; concerns about the data.

## Supplementary Information

**Additional file 1.**

## Data Availability

All data generated or analyzed during this study are included in this published article [and its supplementary information file (Supplementary File_1)].

## Abbreviations

CAT: Catalase
p-JNK: Phosphorylated C-Jun N-terminal kinase
CFA: Complete Freund’s adjuvant
COX-2: Cyclooxygenase-2
DMSO: Dimethyl sulfoxide
ECN: 7β-(3-ethyl-*cis*-crotonoyloxy)-1α-(2-methylbutyryloxy)-3, 14-dehydro-Z-notonipetranone
GSH: Glutathione
GST: Glutathione sulfotransferase
LPS: Lipopolysaccharide
MDA: Malonaldehyde
NO: Nitric oxide
NSAID’s: Non-steroidal anti-inflammatory drugs
NF-κB: Nuclear factor-kappa B
ROS: Reactive oxygen species
RA: Rheumatoid arthritis
SOD: Superoxide dismutase
TLR-4: Toll-like receptor 4
